# A Multiview Deep Learning Method for Brain Functional Connectivity Classification

**DOI:** 10.1155/2022/5782569

**Published:** 2022-10-08

**Authors:** Yu Ji, Cuicui Yang, Yuze Liang

**Affiliations:** Beijing Municipal Key Laboratory of Multimedia and Intelligent Software Technology, College of Computer Science, Faculty of Information Technology, Beijing University of Technology, Beijing, China

## Abstract

The brain functional connectivity classification based on deep learning is a research hotspot nowadays. However, the classification performance is far behind the demand of clinical applications. To alleviate the problem, this paper proposes a multiview deep learning method for brain functional connectivity classification. Firstly, the proposed method adopts multiple brain atlases to identify brain regions and thereby builds different brain functional connectivity of different views. Secondly, it uses a multiview feature selection strategy to select out the most discriminative features of each view with the assistance of other views. Then, it trains a stacked autoencoder to extract deep features of the brain functional connectivity of each view. At last, it utilizes a multiview fusion strategy to take full advantage of complementary information of different views for brain functional connectivity classification. The proposed method has been compared with several deep learning-based brain functional connectivity classification methods on three public datasets of neuropsychiatric disorders. The experimental results have validated the superior performance of the proposed method.

## 1. Introduction

The human brain is an extremely complex system that accomplishes specific tasks through cooperation between brain regions. The cooperation between different brain regions can be represented as the brain functional connectivity (BFC) that is usually obtained by analyzing quantitatively the resting-state functional magnetic resonance imaging (rs-fMRI) data. Previous research indicates that many neuropsychiatric disorders are closely related to the abnormal changes of BFC of the patients [1, 2]. Therefore, research on brain functional connectivity classification (BFCC) has great practical significance as it is helpful to diagnose neuropsychiatric disorders and reveal the pathogenic mechanism of neuropsychiatric disorders.

The existing BFCC methods are mainly divided into two categories—the traditional machine learning-based method and the deep learning-based method. The former uses shallow models to analyze BFC, such as support vector machine (SVM) [2, 3] and least absolute shrinkage and selection operator (LASSO) [4]. Although this method has good performance, it remains to be promoted due to insufficient feature extraction ability caused by its shallow structure. The latter is able to extract BFC features from low levels to high levels, which endows it with stronger feature extraction ability. Stacked autoencoders (SAE) [5, 6] and convolutional neural network (CNN) [7, 8] have become two most popular deep learning modes for BFCC due to their good performance on BFCC. However, facing the BFC data with the high dimension and small sample characteristics, the deep learning-based method still has much room for improvement.

Multiview learning is aimed at studying how to make use of multiview data to build more effective learning models. Due to its effectiveness and universality, multiview learning has received increasing attention in the field of machine learning and data mining. It also has been applied into BFCC of neuropsychiatric disorders. The existing methods usually regard one BFC datum obtained by one brain Atlas as a single-view datum and use different BFC data obtained by different brain atlases to classify neuropsychiatric disorders. For example, Liu et al. [9] extracted multiview feature representations for subjects using multiple brain atlases and performed Alzheimer's disease (AD)/mild cognitive impairment (MCI) classification by SVM. Huang et al. [10] proposed a novel multitemplate ensemble classification framework for autism spectrum disorder (ASD) diagnosis. This framework can automatically allot optimal weight for each template and uses an ensemble classification strategy to get the classification results. Huang et al. [11] also presented a framework to enhance the representation of functional connectivity network by fusing the common and complementary information conveyed in multiple functional connectivity networks. This framework makes use of a multikernel SVM to linearly fuse the selected features from each network for ASD diagnosis. These methods have proved that multiview learning is helpful for improving the performance of BFCC, but they all adopt the traditional machine learning methods.

As the feature extraction ability of deep learning methods is stronger than that of traditional machine learning methods, the performance of BFCC for neuropsychiatric disorders is expected to be further improved if multiview learning is introduced into deep learning-based methods.

Thus, this paper proposes a multiview deep learning method for BFCC (called as MVDL-BFCC). Firstly, the proposed method employs different brain atlases to identify brain regions and constructs different BFCs from multiple views. Secondly, it uses a multiview feature section strategy to pick out the most discriminating BFC features for each view with the help of the information conveyed in other views. Then, it trains a SAE to extract deep features of BFC for each view. At last, it uses a multiview feature fusion strategy to merge the deep features of all views. The innovation of the proposed method is that a multiview feature selection strategy and a multiview feature fusion strategy are introduced into deep learning for BFCC. The two new strategies can comprehensively utilize the complementary information of different views to further improve the performance of deep learning-based method for BFCC. The experimental results have validated the effectiveness of the two new strategies and the superior performance of the proposed method.

## 2. Related Work

BFCC is a kind of computational technology to determine whether subjects have mental disorders by analyzing BFC. In Reference [2], the first method of this kind was proposed. The proposed method used recursive feature elimination (RFE) to select discriminating features and employed a SVM model to distinguish healthy controls from clinically depressed patients. Since then, SVM is widely applied into BFCC. In Reference [3], Khazaee et al. used the graph theory to extract features from BFC and trained a SVM model to classify three groups—healthy controls, MCI, and AD. Wang et al. [12] utilized SVM to distinguish healthy controls from adolescent schizophrenia. Bi et al. [13] pointed out that a single SVM was vulnerable to the kernel function and the penalty coefficient and presented multiple SVMs to classify ASD patients and healthy controls. Besides, LASSO is another popular traditional machine learning method for BFCC. For example, Meszlényi et al. [4] employed dynamic time warping distance to characterize BFC and used LASSO to realize the classification task. In Reference [14], Watanabe et al. proposed a regularization framework where the spatial structure of BFC was explicitly taken into account. The proposed framework used LASSO to perform sparse constraints and utilized SVM to accomplish the classification task. The above methods fully demonstrate that the computational methods based on machine learning are able to realize BFCC. However, their classification performance has much room for improvement due to the fact that they are shallow models based on traditional machine learning and cannot extract deep features.

In recent years, deep learning has become one of the research focuses in the field of BFCC. In Reference [5], Kim et al. adopted the deep neural network (DNN) for BFCC of schizophrenia patients and healthy controls. The proposed method initialized the weights of each hidden layer by SAE-based pretraining and used an adaptive learning algorithm to explicitly control the weight sparsity of each hidden layer via L1 regularization. Li et al. [6] developed a deep transfer learning neural network (DTL-NN) framework for BFCC. The proposed framework firstly trained a stacked sparse autoencoder (SSAE) prototype to learn healthy BFC in an offline learning environment. Then, it transferred the SSAE prototype to a DTL-NN model for a new classification task. In Reference [15], a stacked denoising autoencoder (SDAE) with two hidden layers was trained to extract deep features for identifying ASD patients. The proposed method achieved 70% accuracy in identification of ASD versus healthy controls on the ABIDE dataset. In Reference [16], a SAE was built to distinguish normal aging from MCI, which attained a greater improvement of the prediction accuracy.

CNN is another popular deep learning model for BFCC. Parisot et al. [17] exploited a graph convolutional network (GCN) framework for BFCC. This framework represents each subject as a sparse graph, where its nodes are associated with imaging-based feature vectors, while phenotypic information is integrated as edge weights. Meszlényi et al. [7] built a CNN architecture for BFCC called connectome-convolutional neural network (CCNN). This model can combine information from diverse functional connectivity metrics. Kawahara et al. [8] proposed BrainNetCNN that is a CNN framework to predict clinical neurodevelopmental outcomes from brain networks. BrainNetCNN includes novel edge-to-edge, edge-to-node, and node-to-graph convolutional filters that leverage the topological locality of brain networks. Brown et al. [18] further expanded the BrainNetCNN framework by introducing data-dependent anatomically informed prior regularization terms. Ji et al. [19] developed a new convolutional neural network with element-wise filters (CNN-EW) for BFCC. The proposed method gives a unique weight to each edge of brain network which may reflect the topological structure information more realistically.

Based on the above introduction, it is clear that deep learning has gained increasing attention for BFCC. However, most of the existing studies only make use of single-view BFC data for BFCC. The BFC data from single-view may not fully reflect the characteristics of brain functionality, which would restrict the performance of deep learning for BFCC. Inspired by the recent development of multiview learning, this paper proposes a multiview deep learning method for BFCC.

## 3. Method

### 3.1. Main Idea and Overall Framework

Although BFCC based on deep learning has achieved good performance, there is much room for improvement on how to better utilize the BFC data of the high dimension and small samples' characteristics. The existing deep learning-based methods usually extract deep features from all the brain functional connections. However, all the brain functional connections are redundant for classification since studies have found that a brain disease is related to abnormalities of some functional connections. Thus, feature selection is expected to alleviate dimension disaster and enhance the performance of BFCC. Besides, the existing deep learning-based methods usually exact deep features from BFC obtained by one brain Atlas. In fact, the BFC under different brain atlases can be considered as different organizing ways of functions under different views. Each view of BFC may contain special information that does not exist in the BFC of other views. So it is hopeful to enhance the performance of BFCC by effectively using the complementary information of different views.

Based on the above ideas, this paper proposes a multiview deep learning method for BFCC. As illustrated in Figure 1, the proposed method mainly consists of two parts—the multiview feature selection strategy and the deep neural network learning module with multiview feature fusion. The multiview feature selection strategy is able to select out the most discriminating features of each view under the guidance of complementary information of other views. The selected features of each view are the input of the deep neural network learning module with multiview feature fusion. The selected discriminating features of each view are extracted deep features by an SAE. All the deep features will be fused for classification.

### 3.2. Multiview Feature Selection

To eliminate redundant features and comprehensively use the information of different views, a multiview feature selection strategy is developed. This strategy can pick out the most discriminating features of each view by effectively using complementary information of other views. Detailed description of this strategy is as follows.

Let a training set containing *N* subjects be denoted by *X*={*x*_1_, *x*_2_,…, *x*_*N*_}, where *x*_*i*_ represents the BFC data of subject *i*. Suppose the number of brain atlases that are to locate brain regions for building BFC is *V*. That is, each subject has *V* views of BFC data. Let the dimension of BFC data for view *v* be denoted by *n*_*v*_, thus the dimension of features after concatenating the BFC data of all views is defined by *D*=∑_*v*=1_^*V*^*n*_*v*_. The labels of *N* subjects are expressed as a set. *Y*={*y*_1_, *y*_2_,…, *y*_*N*_}. To make use of the complementary information of different views, all the views are divided into two categories when performing feature selection on the BFC data of view *v*. As illustrated in Figure 2, view *v* is the primary view, while all the other views are auxiliary views.

The multiview feature selection on the BFC data of view *v* is accomplished by the following linear regression model with L1 regularization.

(1) $$\begin{array}{c} \min_{\omega }\frac{1}{2N}\overset{N}{\underset{i=1}{\sum }}{\left\|y_{i}-\omega^{T}x_{i}\right\|}_{2}^{2}+\lambda \overset{2}{\underset{g=1}{\sum }}a_{g}\left\|\omega_{g}\right\|\text{,} \end{array}$$

where *ω* is the *D* dimensional weight vector; *ω*_*g*_ represents the weight vector for the features of different category views, i.e., *ω*_1_ is the weight vector for the features of the primary view, *ω*_2_ is that of the auxiliary views, and they can be concatenated together to form *ω*; *a*_*g*_ denotes the weight coefficient of the weight vector *ω*_*g*_, i.e., *a*_1_ is the weight coefficient of the primary view, *a*_2_ is the weight coefficient of the auxiliary view, and they have the relation. ∑_*g*=1_^2^*a*_*g*_=1.

In the linear regression model with L1 regularization, the L1 penalty term makes most elements of the weight vector *ω* be 0 in the training process. The features corresponding to nonzero elements are considered to be the most discriminative features for classification. The main innovation of the proposed method is the new L1 regularization term that, respectively, assigns different weight coefficients for the primary view and the auxiliary view. A smaller value of *a*_1_ means a smaller punishment on the weight vector of the primary view and a greater punishment on that of the auxiliary view. At this time, there are fewer zero elements in the weight vector of the primary view (*ω*_1_), while there are more zero elements in the weight vector of the auxiliary view (*ω*_2_). Obviously, the new L1 penalty term does not only reduce the data dimension and alleviate the over-fitting phenomenon but also selects out more discriminative features of one view by using complementary information of other views.

In the multiview feature selection model defined in formula (1), the first item is differentiable and the second item is not differentiable. To solve this optimization model, the proximal gradient method is adopted. The objective function defined by formula (1) is decomposed into the following two functions.

(2) $$\begin{array}{c} f\left(\omega \right)=\frac{1}{2N}\overset{N}{\underset{i=1}{\sum }}{\left\|y_{i}-\omega^{T}x_{i}\right\|}_{2}^{2}\text{,}\\ h\left(\omega \right)=\lambda \overset{2}{\underset{g=1}{\sum }}a_{g}\left\|\omega_{g}\right\|\text{.} \end{array}$$

As *f*(*ω*) is differentiable and ∇*f* satisfies the L-Lipschitz condition, there exists a constant *L* that makes the following formula true.

(3) $$\begin{array}{c} {\left\|▽f\left(\omega^{\prime }\right)-▽f\left(\omega \right)\right\|}_{2}^{2}\leq L{\left\|\omega^{\prime }-\omega \right\|}_{2}^{2},\forall \omega ,\omega^{\prime }\text{.} \end{array}$$

Therefore, *f*(*ω*) is approximate to the following equation by Taylor expansion at *ω*_*j*_.

(4) $$\begin{array}{c} \hat{f}\left(\omega \right)\approx \frac{L}{2}{\left\|\omega -\left(\omega_{j}-\frac{1}{L}\nabla f\left(\omega_{j}\right)\right)\right\|}_{2}^{2}+C\text{,} \end{array}$$

where *C* is a constant that is independent of *ω*.

Obviously, the minimum value of the above formula is obtained at *ω*_*j*+1_.

(5) $$\begin{array}{c} \omega_{j+1}=\omega_{j}-\frac{1}{L}\nabla f\left(\omega_{j}\right)\text{.} \end{array}$$

After considering *h*(*ω*), the complete iteration is as follows:

(6) $$\begin{array}{c} \omega_{j+1}={argmin}_{\omega }\frac{L}{2}{\left\|\omega -\left(\omega_{j}-\frac{1}{L}\nabla f\left(\omega_{j}\right)\right)\right\|}_{2}^{2}+h\left(\omega \right)\text{.} \end{array}$$

For the last formula, firstly calculate *ξ*=*ω*_*j*_ − 1/*L*∇*f*(*ω*_*j*_) and then solve the following formula:

(7) $$\begin{array}{c} \omega_{j+1}={argmin}_{\omega }\frac{L}{2}{\left\|\omega -\xi \right\|}_{2}^{2}+h\left(\omega \right)\text{.} \end{array}$$

Let *ω*^*p*^ represent the *p*th component of *ω* and this component correspond to view *g*. If the last formula is expanded, it can be found that there does not exist an item like *ω*^*p*^*ω*^*q*^(*p* ≠ *q*). That is, each component of *ω* does not affect each other. So the last formula has the following closed-form solution:

(8) $$\begin{array}{c} \omega_{j+1}^{p}=\left\{\begin{array}{cc} \xi^{p}-\frac{\lambda a_{g}}{L}\text{,} & if\;\frac{\lambda a_{g}}{L}<\xi^{p}\text{,}\\ 0\text{,} & if\left|\xi^{p}\right|\leq \frac{\lambda a_{g}}{L}\text{,}\\ \xi^{p}+\frac{\lambda a_{g}}{L}\text{,} & if\;\xi^{p}<\frac{\lambda a_{g}}{L}\text{.} \end{array}\right. \end{array}$$

The optimal solution of the objective function defined by formula (1) can be obtained by iterating the formula (8).

After the above optimization process, the obtained feature subset of each view will be served as an input to an SAE for extracting deep features of each view.

### 3.3. Multiview Deep Feature Fusion

Most existing deep learning-based multiview learning methods merely concatenate or add the deep features of each view element by element, as illustrated in Figure 3(a). Although they can obtain deep features from multiple views, they cannot take full advantage of multiview learning without aligning the deep features of each view in the common feature space. To address this problem, a multiview feature fusion strategy is introduced into SAE for merging the deep features of each view. As shown in Figure 3(b), the normalized cross correlation (NCC) between deep features of different views is firstly calculated; then, the normalized cross-correlation is added to the loss function as an regularization item, which can take the role of aligning the deep features of each view in the common feature space.

Next, we take two views as an example to describe in detail the implementation way of multiview feature fusion.  Figure 4 shows how to obtain the first fused deep feature. The calculation ways of other fused deep features are similar. In this figure, *z*=[*z*_1_, *z*_2_,…, *z*_*K*_] represents the fused deep feature vector, where *K* is the number of fused deep features; *v*_1_ and *v*_2_ are two deep feature vectors from two views; *h*=[*v*_1_, *v*_2_] are the concatenated features of *v*_1_ and *v*_2_; *W* is the parameter vector of the feature fusion layer. *u*_1_=[*u*_1_^1^, *u*_1_^2^,…, *u*_1_^*K*^] and *u*_2_=[*u*_2_^1^, *u*_1_^2^,…, *u*_2_^*K*^] are linear transformations of *v*_1_ and *v*_2_, respectively. For *u*_1_ and *u*_2_, their first features are calculated as follows:

(9) $$\begin{array}{c} u_{1}^{1}=w_{1}^{1}v_{1}\text{,}\\ u_{2}^{1}=w_{2}^{1}v_{2}\text{,} \end{array}$$

where *w*_1_^1^ and *w*_2_^1^ are the network parameters corresponding to *v*_1_ and *v*_2_ in the first column of *W*, respectively.

The first feature in the fused deep feature vector *z* is obtained by

(10) $$\begin{array}{c} z_{1}=u_{1}^{1}+u_{2}^{1}\text{.} \end{array}$$

Formula (10) is essentially served as feature extraction by a fully connected layer. To align the fused deep features, maximized correlation of *u*_1_ and *u*_2_ is considered in the model training process. The following normalized cross correlation function is used to measure the correlation of *u*_1_ and *u*_2_.

(11) $$\begin{array}{c} NCC\left(u_{1},u_{2}\right)=\frac{1}{K-1}\frac{\sum_{k=1}^{K}\left(u_{1}^{k}-\mu_{1}\right)\left(u_{2}^{k}-\mu_{2}\right)}{\sigma_{1}\sigma_{2}}\text{,} \end{array}$$

where *μ*_1_=1/*K*∑_*k*=1_^*K*^*u*_1_^*k*^ and *μ*_2_=1/*K*∑_*k*=1_^*K*^*u*_1_^*k*^, respectively, represent the mean values of all features in *u*_1_ and *u*_2_; $\sigma_{1}=\sqrt{\sum_{k=1}^{K}{\left(u_{1}^{k}-\mu_{1}^{k}\right)}^{2}}$ and $\sigma_{2}=\sqrt{\sum_{k=1}^{K}{\left(u_{2}^{k}-\mu_{2}^{k}\right)}^{2}}$, respectively, represent the variances of all features in *u*_1_ and *u*_2_. The value of NCC(*u*_1_, *u*_2_) is between −1 and 1. The closer it gets to 1, the greater the correlation of *u*_1_ and *u*_2_. The closer it gets to −1, the smaller the correlation of *u*_1_ and *u*_2_.

In the model training process, the sum of the normalized cross correlation between deep features of different views is used as a regularization item. Maximizing this term can achieve the alignment of deep features of different views. This term is expressed as

(12) $$\begin{array}{c} L_{MV}=\overset{V}{\underset{v=1}{\sum }}NCC\left(u_{v},u_{v+1}\right)\text{.} \end{array}$$

### 3.4. Classification Model

In the proposed method, the prototype learning is used for classification. The prototype learning classifies instances according to the distance between instances and prototypes. The prototype of each category is initialized to the mean value of extracted features for each category and is defined in the following formula:

(13) $$\begin{array}{c} p_{c}=\frac{1}{N_{c}}\underset{x_{i}\in classc}{\sum }g\left(x_{i}\right)\text{,} \end{array}$$

where *c* ∈ {1,2,…, *C*} denotes a category label; *C* is the number of category; *g*(*x*_*i*_) is the extracted features for the training instance *x*_*i*_.

Given an instance *x*, the Euclidean distance between *g*(*x*) and the prototype of the category *c* is defined as

(14) $$\begin{array}{c} d_{c}={\left\|g\left(x\right)-p_{c}\right\|}_{2}^{2}\text{.} \end{array}$$

The probability that the instance *x* belongs to the category *c* is defined as

(15) $$\begin{array}{c} P\left(y\left|x\right.\right)=\frac{e^{-\gamma d_{y}}}{\sum_{c=1}^{C}e^{-\gamma d_{c}}}\text{.} \end{array}$$

The distance-based cross entropy (DCE) loss is used to measure the classification error.

(16) $$\begin{array}{c} L_{DCE}=-\log\;P\left(y\left|x\right.\right)\text{.} \end{array}$$

Besides, the margin-based prototype (MP) loss is adopted to further improve the generalization ability of the proposed method.

(17) $$\begin{array}{c} L_{MP}={\left(d_{y}-d_{r}+m\right)}_{+}\text{,} \end{array}$$

where d_*y*_ represents the distance of an instance to the prototype of the same category; d_*r*_ represents the minimization distance of an instance to the prototypes of different categories; and *m* is a margin hyper-parameter. The goal of the model training is to reduce the distance of an instance to the prototype of the same category and increase the distance to the prototypes of different categories by minimizing the MP loss.

To sum up, the overall classification loss function is defined as

(18) $$\begin{array}{c} L=L_{DCE}+\lambda_{1}L_{MP}-\lambda_{2}L_{MV}\text{.} \end{array}$$

### 3.5. Algorithm Description

The training process of the proposed MVDL-BFCC method is described in Algorithm 1.

## 4. Experiments and Results

### 4.1. Datasets and Implementation Details

In this section, three common rs-fMRI datasets are used to evaluate the proposed method, including Autism Brain Imaging Data Exchange (ABIDE), Autism Brain Imaging Data Exchange II (ABIDE II), and Attention Deficit Hyperactivity Disorder (ADHD). The three datasets are composed of fMRI data from multiple international institutions around the world. The first two datasets include normal controls and ASD patients. The third dataset consists of normal controls and ADHD patients.  Table 1 shows the subject sizes of different datasets.

All the fMRI datasets are downloaded from the Preprocessed Connectomes Project (PCP) website. Each dataset is firstly preprocessed by configurable pipeline for the analysis of connectomes (CPAC) from PCP. The preprocessing flow includes slice timing correction, motion realignment, normalization, smoothing, nuisance signal removal, band-pass filtering, and registration. Then, a certain number of brain regions in the cerebral cortex by different Atlases are selected as regions of interest. The corresponding mean time-series for each brain region is extracted. After that, the Pearson correlation coefficients (PCC) between each pair of brain regions are calculated to produce an adjacency matrix for each subject. The BFC matrix for each subject is finally obtained by making the Fisher's *z* transformation on its adjacency matrix. The BFC matrix is a symmetric matrix. The upper triangular of this matrix is expanded into vectors in rows to form the feature data of each subject. That is, each subject is represented as a vector of BFC feature. The dimension of this vector is equal to the number of different brain functional connections that are computed as follows:

(19) $$\begin{array}{c} S=\frac{\left(n-1\right)n}{2}\text{,} \end{array}$$

where *n* is the number of brain regions.

In this paper, three brain Atlases are used to produce the multiview data, i.e., CC200 [20], AAL90 [21], and Dosenbach160 [22]. If CC200 is used, each subject is represented as a vector which consists of 200 × (200 − 1)/2=19900 features. If AAL90 is used, each subject is represented as a vector which consists of 90 × (90 − 1)/2=4005 features. If Dosenbach160 is used, each subject is represented as a vector which consists of 160 × (160 − 1)/2=12720 features.

### 4.2. Experimental Setting and Evaluation Indicators

In the experiments, the number of nodes in the first hidden layer is set to 1000 and those in the other hidden layers are set to 100. In the training process, the Adam gradient descent method is used to minimize the loss function. In each iteration, the batch size and the learning rate are set to 96 and 1 × 10^−4^, respectively. To take full advantage of the limited training instances, all the experiments adopt a 5-fold cross-validation. Each dataset is randomly divided into a training set, a validation set, and a testing set in a ratio of 3.1.1.

Five common indicators including accuracy (ACC), sensitivity (SEN), specificity (SPE), positive predictive value (PPV), and negative predictive value (PPV) are used to evaluate the classification performance of the proposed method. These five indicators are, respectively, defined as follows:

(20) $$\begin{array}{c} ACC=\frac{TP+TN}{TP+TN+FP+FN}\times 100\%\text{,}\\ SEN=\frac{TP}{TP+FN}\times 100\%\text{,}\\ SPE=\frac{TN}{TN+FP}\times 100\%\text{,}\\ PPV=\frac{TP}{TP+FP}\times 100\%\text{,}\\ NPV=\frac{TN}{TN+FN}\times 100\%\text{,} \end{array}$$

where TP denotes the number of positive instances that are predicted to be positive instances; TN denotes the number of negative instances that are predicted to be negative instances; FP denotes the number of negative instances that are predicted to be positive instances; FN denotes the number of positive instances that are predicted to be negative instances.

### 4.3. Effects of Multiview Data

To examine the effect of using multiview data, this section constructs three SAE models based on single-view data and four SAE models based on multiview data. The single-view data based SAE models only use one BFC. The multiview data based SAE models use different BFC and concatenate the features of the last hidden layer together for classification. For comparison, all the SAE models have the same settings except the input data.  Table 2 provides the experimental results on the ABIDE I dataset.

From Table 2, it is easy to find that the latter four SAE models that input more than one BFC data have higher classification accuracy than the former three SAE models that input only one BFC data. To be specific, the three SAE models based on two BFC data have a little higher classification accuracy than the former three SAE models based on one BFC datum. The SAE model based on three BFC data obtains the highest classification accuracy and achieves the best performance on three out of five evaluation indicators. These results suggest that different BFCs about different atlases contain complementary information for classification. Besides, a closer look at this table shows that the classification performance is not obviously enhanced with the number of views increasing. This may be because there are a lot of redundant features in the BFC data under different views. Moreover, redundant features would greatly increase with the number of views increasing. To sum up, it is hopeful for further enhancing the classification performance to perform feature selection by determining a proper number of views.

### 4.4. Effects of Multiview Feature Selection

To validate the effectiveness of multiview feature selection on the classification performance, this section sets different weight coefficients for the primary view and the auxiliary view in equation (1). In this equation, *a*_1_ and *a*_2_ represent the weight coefficient of primary view and auxiliary view, respectively. They have the relation. *a*_1_+*a*_2_=1. For them, a bigger value means a greater punishment for the corresponding view and a more sparse weight. When making feature selection on the data of one certain view, the data of the other views should play an auxiliary part. The weight coefficient of the primary view is set to a smaller value, while that of the auxiliary view is set to a bigger value. Thus, more discriminant features of the primary view can be obtained under the guidance of the other auxiliary views.

Figure 5 shows the experimental results. The general trend is that five indicators increase at first and then decrease. When *a*_1_ = 0 and *a*_2_ = 1, the weight coefficient of the primary view is 0, which means no feature selection is carried out on the data. At this time, the classification accuracy is 70.26%. When *a*_1_ = 0.1 and *a*_2_ = 0.9, that is, the weight coefficient of the primary view is 0.1 and the weight coefficient of the auxiliary view is 0.9, all the five indicators enhance except NPV compared with the former case. When *a*_1_ = 0.2 and *a*_2_ = 0.8, three indicators including ACC, SPE, and NPV reach the best results while the rest two indicators rank second. If *a*_1_ goes on increasing, the classification performance would decline on a whole, but it is still better than that without feature selection.

The above results demonstrate that a proper value for the weight coefficient of the primary view helps to sort out more discriminant features from the primary view data by the complementary information of the auxiliary view. A very small value for the weight coefficient of the primary view would pick out more features from the primary view data, but some of which are redundant for classification. Although a too large value for the weight coefficient of the primary view would not select more features from the primary view data, it would pick out more redundant features from the auxiliary view data and still impair the classification performance. According to the experimental results, the best performance is obtained when *a*_1_=0.2. Therefore, *a*_1_=0.2 is used in the comparative experiments.

### 4.5. Effects of Multiview Feature Fusion

The features extracted from different view data can be concatenated or fused in one layer. For example, all multiview features are fused at the last layer and then the fused features are used for classification. All multiview features are concatenated or fused in one middle hidden layer and the fused features are used to further extract deep features for classification. In other words, the position of performing feature fusion has a certain flexibility.

To examine the effect of multiview feature fusion on the classification performance, this section builds six models which have different feature concatenation or fusion ways.  Table 3 gives the experimental results. In this table, *Concat*-*i*(*i*=1,2,3) denotes the model that concatenates all multiview features at the *i*th hidden layer and further extracts deep features from the concatenated features for classification. MvFF-*i*(*i*=1,2,3) denotes the model that fuses all multiview features at the *i*th hidden layer and further extracts deep features from the fused features for classification. It is obvious to see the following two points from this table. (1) The models that adopt multiview feature fusion have better classification performance than that use multiview feature concatenation on the whole. (2) With the number of the hidden layer that performs feature concatenation or feature fusion increasing, the classification performance tends to get better. Based on these two points, MvFE-3 is used in the proposed method, since it has achieved the best performance on four indicators out of five.

### 4.6. Comparative Evaluation

In this section, the proposed method is compared with two traditional machine learning methods and five deep learning methods on three datasets. The two traditional machine learning methods are RFE_SVM [2] and LASSO [4]. The five deep learning methods are BrainNetCNN [9], CCNN [8], SDAE [15], GCN [17], and SAE-PL-DFF [23].

Figures 6–8 show the experimental results. From these figures, it is found that the proposed method obtains the best performance with respect to three evaluation indicators including ACC, SPE, and PPV on the ABIDE I and ABIDE II datasets. As for the remaining two evaluation indicators, the proposed method is slightly inferior to the best method on these two datasets. Moreover, it is exciting to see that the proposed method achieves the best performance with respect to all the evaluation indicators on the ADHD dataset. Based on the above analysis, it can be concluded that the proposed method has a better classification performance on the whole. Therefore, multiview learning can further improve the classification accuracy of the deep learning method for BFCC.

## 5. Conclusion

To further improve the classification performance of the deep learning method for BFCC, this paper proposes a multiview deep learning method for BFCC. The proposed method takes the BFC data from one brain Atlas as a single-view data and uses three different brain atlases to produce multiview BFC data. For the BFC data of each view, the proposed method presents a multiview feature selection strategy to select out the most discriminating features. And then deep features are further extracted by an SAE. Finally, all the deep features of each view are fused for classification by a new feature fusion strategy. The experimental results have validated the superior performance of the proposed method. [24, 25].

The future research is to make use of different modal data to produce richer multiview data to further improve the classification performance.

## Figures and Tables

**Figure 1:** The overall framework of the proposed method.

**Figure 2:** Schematic of primary view and auxiliary views.

**Figure 3:** Two different ways of deep feature fusion. (a) Concatenation and (b) Proposed fusion way.

**Figure 4:** Illustration of multiview feature fusion.

**Figure 5:** Effects of the weight coefficient of the primary view on the classification performance in terms of different indicators. (a) ACC. (b) SEN. (c) SPE. (d) PPV. (e) NPV.

**Figure 6:** Performance comparison of eight methods on the ABIDE I dataset.

**Figure 7:** Performance comparison of eight methods on the ABIDE II dataset.

**Figure 8:** Performance comparison of eight methods on the ADHD dataset.

**Algorithm 1:** The proposed MVDL-BFCC method.

**Table 1:** The subject sizes of different datasets.

Dataset	Normal controls	Patients	Total
ABIDE I	530	505	1035
ABIDE II	487	556	1043
ADHD	418	175	593

**Table 2:** Results of using different views of data on the ABIDE dataset.

Data	ACC (%)	SEN (%)	SPE (%)	PPV (%)	NPV (%)
CC200	69.30	73.60	65.30	68.97	69.90
AAL90	66.78	73.33	59.97	66.17	68.51
Doshen160	67.57	73.64	61.29	66.82	69.57
CC200 + AAL90	69.88	70.32	69.44	70.69	69.18
CC200 + Doshen160	69.84	70.35	69.29	70.67	69.28
AAL + Doshen160	68.64	69.27	67.97	69.44	68.06
CC200 + AAL90 + Doshen160	70.26	71.22	69.27	70.92	70.08

**Table 3:** Results of multiview feature fusion on the ABIDE dataset.

Data	ACC (%)	SEN (%)	SPE (%)	PPV (%)	NPV (%)
Concat-1	70.42	71.81	68.99	70.77	70.27
Concat-2	70.69	71.46	69.81	71.72	69.92
Concat-3	70.92	71.97	69.86	71.53	70.71
MvFF-1	70.81	71.09	70.45	71.77	70.34
MvFF-2	70.93	71.97	69.86	71.53	70.71
MvFF-3	71.19	72.48	69.81	71.84	70.77

## Data Availability

The datasets used to support the findings of this study are available from the corresponding author upon request.
